# Nursing Research on Patients with Chronic Obstructive Pulmonary Disease and Respiratory Failure Based on Big Data

**DOI:** 10.1155/2021/2541751

**Published:** 2021-09-29

**Authors:** Yongqing Chen, Luyi Pan

**Affiliations:** ^1^Department of Respiratory and Critical Care Medicine, Shanghai Chest Hospital, Shanghai Jiao Tong University, Shanghai 200030, China; ^2^Emergency Department, Shanghai Chest Hospital, Shanghai Jiao Tong University, Shanghai 200030, China

## Abstract

This work organically integrates a systematic and individualized nursing plan with big data technology and applies it to the care of patients with chronic obstructive pulmonary disease (COPD) and respiratory failure (RF) and explores the continuous care model based on modern big data technologies to improve COPD and RF. It aims to relieve the symptoms of COPD and RF, reduce the number of acute episodes of COPD and RF and the number of hospitalizations, and improve the quality of life of patients. One hundred COPD and RF patients hospitalized in the respiratory medicine department of a tertiary hospital were selected and were categorized into control and experimental group. The nursing mode of the patients in the control group was the original telephone follow-up in the department, and the contents of the follow-up were determined according to the questions of the patients on the telephone at that time. Based on the original nursing in the department, the experimental group adopted individualized continual nursing plans based on the Internet and big data techniques for patients to conduct a pulmonary rehabilitation-related functional assessment, functional exercise guidance, and health guidance. Experimental results show that, compared with traditional continuous care, individualized continuous care combined with big data techniques can improve the lung function of patients with stable COPD and RF, reduce the number of acute COPD and RF attacks and the number of readmissions, and improve self-management ability and quality of life. The method can be applied and implemented in continuous nursing care.

## 1. Introduction

Chronic obstructive pulmonary disease or COPD is a group of diseases that cause airflow obstruction and breathing-related problems. It includes emphysema and chronic bronchitis. Tobacco smoke is the basic cause of the progression and development of COPD [1]. Exposure to air pollutants in the workplace and environment, genetic factors, and respiratory infections also play a key role in the development of COPD. In the developing world, indoor air quality is thought to play a greater role. Early detection of COPD may change its course and progress [2]. If effective treatment, intervention, and care are not available, acute exacerbations and comorbidities can create a severe impact on the severity of patients' overall disease, which will increase pulmonary heart disease, respiratory failure, and the incidence of clinical emergencies [3]. COPD is a common disease and frequently occurring disease all over the world. Relevant studies have shown that COPD patients account for 8.2% of people over 40 years of age [4]. In addition to the characteristics of high incidence, COPD also has the characteristics of high mortality, poor prognosis, and the patient population is mainly elderly patients, which seriously affects the health and daily life of individuals. The course of COPD is long, and the patients are prone to recurring attacks. It mostly occurs in elderly patients. The disease is divided into acute attack stage and stable stage [5]. Therefore, in clinical treatment, effective and continuous nursing is the key to treating COPD and maintaining a good prognosis [6].

Traditional nursing intervention only includes routine nursing intervention after treatment. Comprehensive nursing intervention based on big data technology has two meanings from the perspective of maximizing the recovery of patients [7–10]. One is to carry out routine nursing interventions, rehabilitation nursing training, health education, mental state assessment, and other nursing interventions for patients in accordance with standardized procedures and rules. The second is to abandon the traditional nursing model, improve nursing management, standardize the overall nursing process and detailed operations, and try to give every patient more suitable nursing. With the development of the Internet and big data techniques, the rapid flow and unification of information have gradually become routine. Therefore, it is necessary to explore the importance of introducing the Internet and big data techniques into the original nursing model [11–13]. Starting from conventional nursing interventions, in recent years, continuous nursing interventions, family nursing interventions, nursing interventions combining Chinese and Western medicine, and nursing interventions based on Internet media and big data have been developed [14, 15]. In developed countries, the more popular nursing modes are continuous nursing intervention and family nursing intervention, and other nursing modes are relatively rare. Based on the unique medical status of China, the patient population is large, the patients and their families lack nursing knowledge, and the nursing awareness after discharge from the hospital is very poor. Therefore, the nursing work is mainly based on conventional nursing intervention. At the same time, due to the rapid development of the Internet in China, continuous care based on the Internet platform has also set off an upsurge [16]. Today, when Chinese medicine is paid more and more attention, integrated traditional Chinese and Western medicine nursing is relatively common and has achieved certain curative effects [17–20]. The use of the Internet and big data to implement comprehensive nursing interventions is more flexible and convenient in terms of process improvement, operation standardization, and nursing communication.

The rest of the paper is organized as follows: In section 2, related work on COPD and RF is presented. In section 3 the proposed method is discussed. In section 4, experimental results are presented, and finally in section 5, the conclusion is given.

## 2. Related Work

Scientific nursing has practical application in reducing the number of hospitalizations, readmission rate, and medical economic burden and improving the quality of life [21]. Subsequently, nursing received a deeper level of attention and development and gradually became a systematic nursing model [22]. In China, continuity care was introduced by Hong Kong and Taiwan researchers. The initial research focus was mainly on chronic diseases such as diabetes, chronic kidney disease, and COPD, and good results were achieved [23]. With the increasing medical requirements of patients, continuity care has been paid more attention in the mainland [24].

The rapid development of the Internet has brought new opportunities for all walks of life. The organic integration of the Internet with different industries has become a development aspect in recent years. The application of the Internet in health care has created a new medical information service model. In developed countries, it has become more common to develop medical services through Internet platforms and new media technologies [25–27]. To maximize the use of limited medical resources, there is an urgent need to develop health-related information and communication techniques to provide patients with more cost-effective medical and healthcare services [28]. Nursing based on big data and the Internet has been one of the hot spots in nursing research in recent years. The organic integration of big data and nursing is still content that needs in-depth research. The application of big data in continuity care can be divided into four categories: communication software, application, network platform, and hospital-community management network. Nursing based on communication software is currently the most basic and most commonly used method. Foreign Wiseman and others communicate with patients through mobile phone chat software and implement continuation care of postoperative wound rehabilitation for postoperative patients [29]. Communication software such as WeChat and QQ is relatively popular in my country and is widely used in nursing. Wang [30] established a WeChat group for health education so that patients discharged from the hospital after thyroid cancer have the knowledge to reduce the occurrence of adverse events. Ye et al. [31] used the establishment of QQ groups and WeChat groups to conduct community family management of diabetic patients, guide the monitoring of blood sugar, formulate diabetic diet, and supervise exercise, which improved the self-management ability and treatment compliance of diabetic patients. APP-based care is more systematic and professional, but its development cost is higher. Some foreign researchers have developed a mobile health APP for patients with COPD [32], which is divided into modules for health education and disease management for patients. Based on the continuous care of the network platform, through various medical and health websites, patients can obtain health-related information and different levels of health guidance. In foreign countries, more people combine remote monitoring technology with network platforms to discover patients' conditions in time and reduce the occurrence of adverse events [33]. Vinitha et al. [34] developed a machine learning decision treemap algorithm by using structured and unstructured data from the hospital. It also used the map-reduce algorithm for partitioning the data. Compared with several typical calculating algorithms, the scheming accuracy of their model was higher in terms of prediction accuracy. Ram et al. [34] designed a novel technique to use various data sources for forecasting the number of asthma-related emergency department visits. The system acquired data from Twitter and environmental sensors to detect the number of asthma emergency department visits. Dequan et al. [35] developed a Mayo Clinic healthcare system to collect and store enterprise data. It performs analysis of clinical data for diagnosis, treatment, and clinical reporting. Alexandra et al. [36] described the challenges associated with machine learning approaches in the big data platforms and reported that the machine learning methods are best suitable for the prediction of challenges in big data analytics. Min et al. [37] proposed a CNN-based multimodal disease risk prediction algorithm for healthcare data. The algorithm was effective for the disease analysis healthcare community. In this study, we introduce the Internet and big data techniques into comprehensive nursing intervention, which is representative and epoch-making. Experimental results show that the proposed technique can improve the lung function of patients with stable COPD and RF, reduce the number of acute COPD and RF attacks and the number of readmissions, and improve self-management ability and quality of life.

## 3. Methods

In this work, the nursing research on patients with chronic obstructive pulmonary disease and respiratory failure based on big data is conducted. The overall architecture of the proposed nursing care process is illustrated in Figure 1.

### 3.1. Research Objects

Patients who were hospitalized in the department of respiratory medicine of a tertiary hospital from January 1, 2018, to April 1, 2018, were diagnosed with COPD. Guidelines for the diagnosis and treatment of COPD were as follows.

#### 3.1.1. Clinical Manifestations

*Symptoms*. All those patients were selected having characteristic symptoms of chronic and progressively worsening dyspnea, cough, and sputum production. Common symptoms included dyspnea, chronic cough, sputum production, wheezing, and chest tightness and were accompanied by systemic symptoms such as weight loss and loss of appetite.

*Medical History*. Patients having a history of exposure to risk factors and other respiratory diseases in the past, the prevalence season was more than the cold season of autumn and winter, and there was a history of recurring respiratory infections, and patients with a history of pulmonary heart disease were also selected.

*Signs*. Although there may be no obvious signs of COPD in the early stage. As the disease progresses, abnormalities of the thoracic shape such as barreled chests often appear, and shallow breathing, rapid breathing, breathing in a forward sitting position, auscultation revealing low nonbreath sounds, and prolonged breathing also appear. Patients having all of the mentioned signs were also included.

#### 3.1.2. Laboratory Examinations and Other Test Indicators

*Lung Function Test*. To determine the persistence of airflow limitation, a lung function test was performed for patients.

*Chest X-Ray Examination.* Although there may be no obvious changes at the beginning of the period, however, after sometimes, increased lung texture may appear, which is an indication of COPD.

*Chest CT Examination*. This test is used to distinguish it from other diseases.

*Pulse Oxygen Saturation Monitoring and Blood Gas Analysis*. This test is applied to determine whether there is respiratory failure.

*Differential Diagnosis*. It helps distinguish it from asthma, bronchiectasis, cardiogenic heart failure, and bronchitis. The entire research process follows the inclusion and exclusion criteria.

*Inclusion Criteria.* Diagnosed as chronic obstructive pulmonary disease, in line with the diagnostic criteria in the 2013 “Chronic Obstructive Pulmonary Disease Diagnosis and Treatment Guidelines”; after treatment, the course of the disease is in a stable phase, consistent with the 2013 “chronic obstructive pulmonary disease diagnosis and treatment guidelines.” The standard of the period is that the patient's COPD symptoms are stable or the symptoms are mild, and the condition returns to the state before the acute attack. The age is less than 65 years, the lung function is graded from mild to severe, and the patient is clear and can read and speak. Communication with medical staff is barrier-free, and patients and their caregivers have the habit, conditions, and ability to use the Internet and can use smartphones proficiently. If they know the content of the research, they volunteer to participate in this research.

*Exclusion Criteria*. Patients with mental disorders and disturbances in consciousness or mobility; patients with other cardiovascular diseases, kidney damage, liver damage, or neurological diseases; patients with other severe lung diseases, such as interstitial pneumonia, lung malignancy tumor, bronchial asthma or chest, and lung surgery, combined with infectious respiratory diseases such as tuberculosis, combined with bacterial pneumonia, living in a remote area, unable to carry out on-site follow-up; and those participating in other similar experimental studies were excluded.

*Termination Criteria.* The study should be withdrawn if the following circumstances occur during the study: the subject asks to withdraw; during the study, the patient automatically withdraws due to objective reasons such as disability, death, and infectious respiratory disease, the patient and his direct care patients cannot follow up as planned. Other researchers believe that continuing to participate in the study may cause adverse consequences to the patients or their caregivers.

### 3.2. Intervention Nursing Based on Big Data

In the hospital, general data surveys were conducted on the subjects of the experimental group, and the general data questionnaires were drawn up by the researchers themselves. When the patient's condition entered a stable phase and was ready to be discharged, the experimental group of patients was evaluated based on baseline data, that is, the preliminary assessment. The CAT scale was used to evaluate the patient's disease symptoms, and the lung function test was used to evaluate the patient's airflow limitation. We also employed the SGRQ-C questionnaire to evaluate the patient's quality of life and used the CDSMS scale to evaluate the patient's self-management ability.

Upon discharge from the hospital, the nurse established a WeChat connection with the patient and their direct caregivers to establish a COPD continuing care WeChat exchange group. At the same time, the nurse establishes a separate WeChat connection with each patient and their direct caregivers. The nurse maintained an electronic file for each patient. The file content included basic patient information, initial evaluation results, individualized continuation care plan, staged evaluation results, and final evaluation results.

According to the big data-based nursing program, health education was provided to patients, including online and offline missions. Online education means that nurses use big data techniques to make the content of the education into an appropriate form and use big data platforms such as WeChat to push it. Online publicity and education are regularly pushed according to the needs of patients. At the same time, real-time online replies and irregular assessments were used to ensure that patients and their direct caregivers can effectively read, browse, and learn to push content. The form of offline education was family visits, and on-site guidance was provided according to the needs of patients. The content of health education included the following.

*Functional Assessment*. To improve the patients and their direct caregivers' understanding of COPD and their ability to deal with the disease self-disease function assessment can help patients grasp the level of lung function, exercise endurance, and health status, then understand and judge the progress of the disease, and understand the timing of visits to the doctor.

*Rehabilitation Exercise*. This exercise can be divided into endurance training, resistance training, and breathing training. Endurance training can improve the ability of aerobic exercise through exercise and then improve the function of peripheral muscles. Endurance training is dominated by aerobic exercise. Resistance training is divided into upper extremity training and lower extremity training. The upper extremity training methods include chest expansion exercises, arms raising exercises, back extension exercises, ball gripping exercises, pulley exercises, and height touch exercises. The resistance training intensity should not aggravate the patient's dyspnea. The specific plan depends on the patient's condition. The principle of resistance is gradual, paying attention to relaxation and stretching of the limbs. The purpose of breathing training is to improve the strength and coordination of the respiratory muscles by establishing an effective breathing method. According to the individualized big data nursing plan, the nurse prepares the rehabilitation exercise plan for the patient, including exercise method, exercise duration, and exercise frequency. Nurses train patients and direct caregivers in rehabilitation exercise skills as well as supervise and evaluate the rehabilitation exercise process.

*Guidance on Disease-Related Knowledge*. Online education is for nurses to take pictures, articles, and videos of disease knowledge education and push them to patients and their families through big data platforms. In addition, nurses establish online patient groups. Offline education mainly refers to family visits, where nurses enter the patient's home, provide psychological counseling to the patient and their direct caregivers, and answer questions about disease-related knowledge.

*Home Oxygen Therapy and Noninvasive Ventilator*. COPD patients with dyspnea accompanied by hypoxemia can be given home oxygen therapy; instruct patients to use nasal catheters; continuous low-flow oxygen inhalation, oxygen therapy, and ventilator use-related online education of knowledge is mainly to push operation videos and precaution articles to patients and their direct caregivers; and ask patients and their direct caregivers to shoot daily use processes as videos and upload them so that nurses can spot check, find errors, and provide guidance. Offline education is the correct way for nurses to guide the on-site installation, removal, cleaning, and maintenance of the ventilator during home visits.

*Medication Guidance.* Inhalation therapy is the focus of drug therapy for patients with stable COPD. Doctors and nurses jointly recommend individualized inhalation devices for patients based on evaluation, cost, prescription, and the ability and preferences of patients. Demonstration and training of inhalation devices were provided by nurses to patients and their direct caregivers. Online education is where nurses push videos of inhalation operations, pictures of decomposition actions, articles on adverse drug reactions through the WeChat platform, calling on patients and their direct caregivers to learn, and at the same time encouraging patients and their direct caregivers to upload their usage. Nurses can conduct spot checks. Offline guidance is the on-site guidance and demonstration of the correct use of inhalants when nurses are visiting at home.

Besides, this article evaluates the nursing plan based on big data from the following aspects:

- When in the hospital, nurses assess the requirements of patients through the data questionnaire and guide the key contents of the individualized big data nursing plan.
- Upon discharge from the hospital, perform an initial assessment of each patient.
- For functional assessment, the nurse will perform a CAT assessment on the patient when discharged from the hospital, and the nurse will ask and record the patient's self-CAT assessment every week when out of the hospital. At monthly home visits, the nurse will assess whether the patient and their direct caregivers are using the CAT correctly.
- Regarding rehabilitation exercises, after discharge from the hospital, nurses will conduct an assessment after training the patient and the patient's direct caregivers to assess the patient and his direct caregivers' mastery of rehabilitation exercise skills. After health education, the nurse will regularly check the completion progress of the patient's rehabilitation exercise plan, spot check the patients and their direct caregivers to upload exercise videos to evaluate the practice status of the patients and their direct caregivers, and monthly home visits to evaluate the patient's rehabilitation exercise correctness.
- Regarding disease-related knowledge, the nurse will assess the disease-related knowledge of patients and their direct caregivers through the WeChat platform from time to time and evaluate their mastery of the content of publicity and education.
- For home oxygen therapy and noninvasive ventilator, after discharge from the hospital, nurses demonstrate the use of home oxygen therapy and noninvasive ventilator. When family members and their direct caregivers use it by themselves, the nurse also evaluates whether their use is standardized and correct. Outside the hospital, the nurse randomly checks the videos uploaded by patients every week to assess whether their use is standardized and correct. Conduct on-site assessment during monthly home visits.
- For medication guidance, after the nurse demonstrates the inhaler when discharged from the hospital, assess whether the patient has accurately grasped the correct use of the inhaler. Outside the hospital, through weekly online videos, assess whether the patient's inhalation is used correctly and whether it is in compliance with the doctor. The nurse conducts on-site assessments through monthly home visits.
- After 6 months, a retest evaluation will be conducted, including symptoms, lung function, quality of life, self-management ability, number of readmissions within six months, and patient satisfaction.

### 3.3. Statistical Method

All the data in this study were statistically analyzed using SPSS22.0 statistical software. In the general data of the research subjects, the counting data are expressed as frequency and composition ratio (%), and the measured data are expressed as mean ± standard deviation. The general data comparison between the control group and the experimental group adopts chi-square analysis, and the age data adopt *t*-tests. Among the measurement indicators of the study subjects, the measurement data are expressed as mean ± standard deviation. The measurement indicators of the two groups of patients are compared by *t*-tests, and the comparison of measurement indicators before and after the intervention is by paired *t*-tests. The test level of all statistical tests in this study is *α* = 0.05, and the difference is considered statistically significant when *P* < 0.05.

## 4. Experimental Results and Analysis

### 4.1. CAT Score before and after Intervention

The computer adaptive testing (CAT) scores of the two groups of patients met a normal distribution, and the *t*-test is used for comparison between the two groups of patients before and after the intervention. The CAT scores before the intervention were 12.30 ± 4.11 points for the control group and 12.94 ± 4.15 points for the experimental group, both of which belonged to a moderate impact. There is no statistically significant difference in the CAT scores of the two groups before the intervention (*P* > 0.05). After the intervention, the CAT scores of the control group and the experimental group are 10.87 ± 5.67 points and 9.18 ± 6.33 points, respectively. After the intervention, the CAT scores of the two groups are reduced compared with those before the intervention. The difference within the group is statistically significant (*P* < 0.05). Comparing the two groups of patients after the intervention, the CAT score of the experimental group is lower than that of the control group, and the difference is not statistically significant (*P* > 0.05). The detail is given in Table 1 and Figure 2, where CG represents the control group and EG represents the experimental group.

### 4.2. Pulmonary Function Indexes before and after Intervention

The lung function test results of the two groups of patients before and after nursing all satisfy the normal distribution. Before and after the intervention, the lung function FEV1/FVC (%) index of the two groups is compared by the *t*-test. The results show that the lung function of the experimental group is better than that before the intervention. The relevant indicator FEV1/FVC (%) in the control group and the experimental group before the intervention is 55.97 ± 5.95 and 56.98 ± 6.59, respectively. There is no statistically significant difference between the two groups of patients before intervention (*P* > 0.05). The related indexes of lung function after intervention are 55.66 ± 5.20 in the control group and 59.88 ± 6.13 in the experimental group. Pulmonary function test results of the two groups of patients before and after intervention are compared by the paired *t*-test. The results show that the lung function indexes of the control group changed little before and after the intervention, and there is no significant change in FEV1/FVC (%). This shows that there is no significant difference in comparison within the group (*P* > 0.05). The lung function indexes of the experimental group after 6 months of nursing based on big data are significantly increased than that before, and the differences within the group are statistically significant (*P* < 0.001). After nursing, the indexes of the experimental group are higher than those of the control group. The difference between the groups is statistically significant (*P* < 0.05). The results are shown in Table 2 and Figure 3.

### 4.3. Quality of Life before and after Intervention

The SGRQ-C scores of the two groups of patients met a normal distribution. The initial SGRQ-C scale score of the control group is 64.55 ± 7.08 points, and the initial SGRQ-C scale score of the experimental group is 65.42 ± 6.26 points in total. The scores of all dimensions of the patients in the group are consistent with the total scores, and the quality of life of the two groups of patients before the intervention is at the middle to a low level. The total scores of SGRQ-C and the scores of each dimension of the two groups of patients before and after the intervention are compared by the *t*-test. The initial SGRQ-C total scores and scores of each dimension of the two groups are compared between the groups, and the difference is not statistically significant (*P* > 0.05). The life score of the control group after the intervention is 55.99 ± 16.87 points, and the score of the SGRQ-C scale of the experimental group after the intervention is 45.48 ± 18.12. A paired *t*-test was used to compare the two groups of patients before and after the intervention. The results show that the total score of SGRQ-C in the control group is lower than that before the intervention. The difference within the group is statistically significant (*P* < 0.05). After the intervention, the scores between the groups are lower than those of the control group, and the differences between the groups are statistically significant (*P* < 0.05). The results are shown in Table 3 and Figure 4.

### 4.4. The Number of Hospital Admissions and Satisfaction after Intervention

After 6 months, the number of readmissions within six months of the control group is 1.17 ± 0.75, and that for the experimental group is 0.58 ± 0.71. The number of readmissions within six months of the experimental group is less than that of the control group, and the test result is statistically significant (*P* < 0.05). The satisfaction score of the control group is 77.74 ± 8.15 points, and that of the experimental group is 86.55 ± 4.67 points. It is evident that the satisfaction score of the experimental group is higher than that of the control group. The difference between the groups is statistically significant (*P* < 0.001). The details of this experimental process are given in Table 4, where RH represents several rehospitalizations.

## 5. Conclusion

Compared with conventional nursing methods, according to the individual needs of patients with stable COPD, in this study, a multidisciplinary medical collaboration model is used to comprehensively evaluate patients. Patients with COPD and RF disease were selected and were categorized into control and experimental groups. The nursing mode of the patients in the control group was the original telephone follow-up in the department, and the contents of the follow-up were determined according to the questions of the patients on the telephone at that time. The experimental group adopted continual nursing plans based on the Internet and big data techniques for patients to conduct a pulmonary rehabilitation-related functional assessment, functional exercise guidance, and health guidance. This mode of nursing care improved the clinical symptoms and lung function of patients with stable COPD, improved the quality of life, reduced the number of readmissions, and increased patient satisfaction. Moreover, this kind of continuity nursing model research is better than traditional continuation nursing for patients with stable COPD, and it is worthy of clinical promotion.

## Figures and Tables

**Figure 1:** The architecture of research design for nursing is based on big data.

**Figure 2:** Comparison of CAT scores before and after the intervention (^*∗*^represents *P* value less than 0.05, and ^*∗∗*^represents *P* value less than 0.001).

**Figure 3:** Comparison of FEV1/FVC scores before and after the intervention (^*∗*^represents *P* value less than 0.05, and ^*∗∗*^represents *P* value less than 0.001).

**Figure 4:** Comparison of life quality before and after the intervention (^*∗*^represents *P* value less than 0.05, and ^*∗∗*^represents *P* value less than 0.001).

**Table 1:** Comparison of symptoms before and after intervention (CAT).

Item	Intervention	CG	EG	*T*	*P*
CAT	Before	12.30 ± 4.11	12.94 ± 4.15	−0.68	0.57
	After	10.87 ± 5.67	9.18 ± 6.33	1.26	0.23

**Table 2:** Comparison of pulmonary function before and after the intervention.

Item	Intervention	CG	EG	*t*	*P*
FEV1/FVC	Before	55.97 ± 5.95	56.98 ± 6.59	−0.59	0.59
	After	55.66 ± 5.20	59.88 ± 6.13	−3.17	0.002

**Table 3:** Comparison of life quality before and after the intervention.

Item	Intervention	CG	EG	*t*	*P*
FEV1/FVC	Before	64.55 ± 7.08	65.42 ± 6.26	−0.43	0.72
	After	55.99 ± 16.87	45.48 ± 18.12	2.53	0.017

**Table 4:** Comparison of life quality between the groups after the intervention.

Item	Intervention	CG	EG	*t*	*P*
RH	After	1.17 ± 0.75	0.58 ± 0.71	3.52	<0.001
Satisfaction	After	77.74 ± 8.15	86.55 ± 4.67	−5.99	<0.001

## Data Availability

The data sets used and/or analyzed during the current study are available from the corresponding author on reasonable request.
